The article "Safety and Efficacy of Single Condylar Knee Prosthesis When Treating Knee Single Compartment Osteoarthritis: A Prospective, Case-Randomized Controlled Study" was published in 2022. Journal: Comput Intell Neurosci.

# Safety and Efficacy of Single Condylar Knee Prosthesis When Treating Knee Single Compartment Osteoarthritis: A Prospective, Case-Randomized Controlled Study

**DOI:** 10.1155/2022/3722619

**Published:** 2022-07-30

**Authors:** Shaofeng Wang, Yang Wang, Jiong Wang

**Affiliations:** ^1^Department of Orthopedics, Jinshan Tinglin Hospital, Shanghai 201505, China; ^2^Department of Orthopedics, Seventh Medical Center of PLA General Hospital, Beijing 100700, China; ^3^Department of Orthopedics, Caidian District People's Hospital, Wuhan 430100, Hubei Province, China

## Abstract

**Objective:**

The aim of this study is to explore the safety and efficacy of single condylar knee prosthesis when treating knee single compartment osteoarthritis by measuring the decrease of hemoglobin, total postoperative blood loss, maximum reduction of HCT, and knee joint activity.

**Methods:**

A total of 80 patients with knee joint single compartment osteoarthritis treated in our hospital from January 2020 to December 2021 were studied. They were randomly assigned to a study group (*n* = 40) and a control group (*n* = 40). The study group was treated with total knee prosthesis, while the control group was treated with simple knee prosthesis. The decrease rate of hemoglobin, the amount of bleeding, and the maximum decrease of hematocrit were compared after treatment. The range of motion of knee joint was evaluated by the Fugl-Meyer motor function scale (FM-B) and Berg balance scale (BBS).

**Results:**

The decrease of hemoglobin in the study group at 24 hours, 36 hours, and 48 hours after treatment was remarkably lower (*P* < 0.05). The total blood loss and the maximum reduction of hematocrit(HCT) in the study group were lower (*P* < 0.05). The range of motion (ROM) of the knee joint in the study group at 6 and 12 months after treatment was remarkably higher than that before treatment and remarkably higher compared to the control group (*P* < 0.05). The FM-B scale and BBS scale of the studied cohort at 6 and 12 months after treatment were remarkably higher than those before treatment and were remarkably higher compared to the control's (*P* < 0.05).

**Conclusion:**

The unicondylar knee prosthesis is safer and more effective in the treatment of noncompartmental osteoarthritis of the knee, facilitating less trauma and perioperative blood loss and enhancing the patient's motion and balance.

## 1. Introduction

Knee joint single compartment osteoarthritis (single-compartment osteoarthritis of the knee joint) is an obvious bone and joint disease [1]. The disease shows chronic progression and the pathology is dominated by noninflammatory changes, such as articular cartilage degeneration and secondary hyper osteogeny. The disease mostly occurs in the middle-aged and elderly accompanied with the increasing age of prevalence rate, and the incidence rate in female is higher than that in male [2, 3]. The main clinical symptoms are joint pain, stiffness, swelling, and limitation of movement, which bring great pain and inconvenience to the patients' life and work.

The article "Safety and Efficacy of Single Condylar Knee Prosthesis When Treating Knee Single Compartment Osteoarthritis: A Prospective, Case-Randomized Controlled Study" was published in 2022. Journal: Comput Intell Neurosci.

Anatomically, the knee joint can be assigned into three compartments, including medial compartment, lateral compartment, and patellofemoral compartment. Knee arthritis can affect any of these compartments and damage to any compartment can lead to loss of knee joint function [4]. Clinically, the early pathological changes in patients with 1/3 were limited to one compartment, in which the medial compartment was more common, and the lateral intercompartment and patellofemoral compartment were rarely involved [5, 6]. The early stage of knee osteoarthritis is mainly a mild dull pain in the part of the knee, which is often aggravated after activity and proper rest may be relieved. However, as the disease progresses, the symptoms will become more and more serious [7–9].

At present, orthopedic clinic has a variety of step-by-step treatment for knee osteoarthritis at different stages of development [10]. The surgical methods for the treatment of single compartment osteoarthritis include total knee arthroplasty and single condylar replacement. Total knee arthroplasty as a clinical near-perfect treatment for advanced knee osteoarthritis, its long-term postoperative survival rate and excellent and good rate have basically been recognized by most scholars [11, 12]. However, because the human knee joint is unique in its own structure and lower limb force line, there are not a few knees osteoarthritis manifested by unilateral compartment in clinic, mainly the medial knee compartment as the mainstream. It accounts for about half of all patients with knee osteoarthritis. However, at present, for some patients with medial compartment, whether it is suitable for direct total knee arthroplasty, there are still objections at home and abroad [13–15]. For this reason, as early as the late 1960s, some scholars had proposed a surgical treatment for single compartment osteoarthritis of the knee joint, which was called single condylar replacement [16]. Single condylar knee prosthesis replacement preserves the relatively healthy knee compartment of the patient through the compartment replacement of the knee joint lesion of the patient. After more than half a century of development, a surgical technique has been gradually improved and perfected. Compared with total knee arthroplasty, it has the advantages of small incision, nonvalgus patella, preservation of quadriceps femoris, no interference with suprapatellar bursa and extension device, less trauma, and early weight bearing after operation. This operation retains as much normal bone and soft tissue as possible, causing less surgical trauma to patients, and the time of the operation is relatively shorter. It has even become the last surgical treatment for some patients with knee osteoarthritis. Therefore, a prospective, case-randomized controlled study was conducted to study the safety and efficacy of unicondylar knee prosthesis when treating knee single compartment osteoarthritis.

The article "Safety and Efficacy of Single Condylar Knee Prosthesis When Treating Knee Single Compartment Osteoarthritis: A Prospective, Case-Randomized Controlled Study" was published in 2022. Journal: Comput Intell Neurosci.

## 2. Patients and Methods

### 2.1. General Information

Eighty patients (80 knees) with knee joint single compartment osteoarthritis who were cured from January 2020 to December 2021 were enrolled in our hospital as the subjects of the study. The 80 patients were arbitrarily assigned into studied and controlled groups. There were 40 cases (40 knees) in the study group and 40 cases (40 knees) in the control group. 20 males and 20 females were in the research cohort, who aged from 48 to 64 years old (mean age 55.36 ± 4.22). There were 21 cases of right knee and 19 cases of left knee. 21 males and 19 females were in the controlled cohort, who aged from 48 to 65 years old (mean 53.42 ± 4.17). The lesions were located in the right knee in 21 cases and the left knee in 19 cases. There exhibited no significant difference in sex, age, and course of disease.

The inclusion criteria of this study are as follows:

1. The anterior and posterior cruciate ligaments and the medial and lateral collateral ligaments were normal.
2. The symptoms of pain or tenderness in the medial compartment of the knee joint are obvious, but there were no obvious symptoms in other compartments.
3. Weight-bearing standing knee X-ray showed that the medial compartment had osteoarthritis manifestations of grade III-IV by Kellgren–Lawrence (K–L) classification, and other compartments were normal or had no imaging manifestations of grade III or above.
4. There was no varus and valgus deformity of knee joint or varus ≤15°. The deformity could be corrected by manipulation.
5. Flexion deformity <15°, ROM ≥90°.

The exclusion criteria of this study are as follows:

1. Patients with abnormal blood coagulation found by laboratory examination.
2. The patient had recently or is currently using some kind of an anticoagulant.
3. Patients with ischemic heart disease or chronic cardiac insufficiency, atrial fibrillation, and stent implantation.
4. Patients with previous history of thrombosis and cerebral infarction.
5. Patients with active infection.
6. Patients with severe cardiac and pulmonary insufficiency; patients with liver insufficiency (pay special attention to patients with low albumin), patients with renal insufficiency.
7. Patients with hemoglobin <90 g/L or with other hematological disorders.
8. Unable to complete the research for various reasons.

The article "Safety and Efficacy of Single Condylar Knee Prosthesis When Treating Knee Single Compartment Osteoarthritis: A Prospective, Case-Randomized Controlled Study" was published in 2022. Journal: Comput Intell Neurosci.

### 2.2. Treatment Methods

#### 2.2.1. Technical Route

The technology roadmap is as indicated in Figure 1.

#### 2.2.2. Treatment Scheme

After a clear diagnosis was made, the patient and his or her family agreed to or requested artificial joint replacement treatment. The patients needed to complete the necessary perioperative tests to exclude inappropriate factors. The patients then underwent elective surgery.

The operation plan of the control group: total knee joint surface prosthesis replacement: after anesthesia was effective, a supine position was taken, catheterization was normal, routine disinfection area, sterile sheet, and a protective film was routinely applied in the operation area. The thighs were preset with an inflatable tourniquet. A straight anterior incision of the knee was taken, about 10–12 cm, bended the knee and valgus the patella. During the operation, it was common to see the injury of the cartilage surface of femur, tibia, and patella, the formation of peripheral osteophyte, synovial hyperemia, hyperplasia and hypertrophy, removal of hyperplastic synovium, residual meniscus and anterior and posterior cruciate ligament, and removal of osteophyte and loose body. According to the biological force line of the lower limb, the tibial plateau, anterior and posterior condyle of femur, distal end, oblique plane, and groove were cut to repair the articular surface of patella. After patella shaping, the corresponding test model, flexion, and extension joint, joint stability, ROM, force line, and patellar trajectory were all satisfactory. Then, the joint prosthesis was gradually implanted into the knee joint with bone cement. Burn gauze pressure bandaging, no drainage tube after the operation, total knee joint surface prosthesis replacement side prosthesis-enrolled Zimmer NexGen knee joint prosthesis, the operation was performed by the same group of surgeons.

Operation plan of the research group: After the effect of anesthesia, the patients were taken in a supine position, normal indwelling catheterization, routine disinfection area, aseptic sheet, upper limb driving belt and tourniquet, and a protective film was routinely applied in the operation area. A 10 cm incision was made longitudinally on the medial line of the patella of the affected knee. The skin, subcutaneous tissue, and fascia were cut layer by layer and the joint capsule was cut in the medial side of the patella. The osteophyte at the edge of the femoral condyle and tibial plateau were removed, and the soft tissue appropriately was released. If necessary, it was checked whether there were lesions on the cartilage surface of the patella, the articular surface of the lateral compartment cartilage and whether the cruciate ligament was normal. Finally, the surgical indications were confirmed. The external positioning rod of tibial bone marrow was installed to locate the osteotomy. The positioning rod in the femoral bone marrow was inserted to determine the location of osteotomy and then osteotomy. The tibial plateau prosthesis was installed, and the knee joint was flexed and extended to test the stability of the knee joint and the tension of the surrounding soft tissue. The femoral prosthesis was installed to test the model, fully flexion, and extend the knee joint to ensure that the movement of the patella would not be hindered during flexion and extension. The bone surface was rinsed, the bone cement was mixed, the tibia prosthesis and femur prosthesis were placed in turn, the excess bone cement was scraped off, the bone cement was pressed to harden completely, and the knee joint was kept to the neutral position during the period. Bite forceps to repair the osteophyte around the patella. The placement of high polyethylene gasket, full flexion, and extension of the knee joint can carry out a sufficient range of activities. Patellar movement trajectory was normal without hindrance. The drainage tube was retained, the drainage device was connected, and the incision was sutured layer by layer. OxfordPhase3 knee prosthesis made by Biomet Company was enrolled for unicondylar knee prosthesis replacement and all the operations were performed by the same group of surgeons.

The article "Safety and Efficacy of Single Condylar Knee Prosthesis When Treating Knee Single Compartment Osteoarthritis: A Prospective, Case-Randomized Controlled Study" was published in 2022. Journal: Comput Intell Neurosci.

The blood routine, ion routine, ESR and C-reactive protein, and the positive and lateral position of knee joint X-ray were examined after operation. The drainage tube was removed when the drainage volume was less than 100 ml within 48 hours. The antibiotics were used to prevent infection if necessary. Subcutaneous injection of enoxaparin sodium (4000iu, once a day) was given on the first day after operation and rivaban (10 mg, once a day) was taken orally from the second day to 5 weeks after operation.

Active quadriceps contraction exercises, ankle flexion and extension exercises, and straight leg raising exercises were carried out on the first day after operation. Knee flexion and extension exercises and walker-assisted weight-bearing walking were carried out on the second day after operation and gradually increased the range of flexion and extension of the knee joint and full weight-bearing walking according to the situation. On the first day after operation, 5 kg weights (rice bags or salt bags) were placed on the knee joint after operation and straightening exercises were carried out until the knee joint could straighten itself. The dressing was changed regularly and the healing of the incision was observed. The patients with good incision healing, no fever, no infection, knee joint reached 0° extension position 90° flexion position can be discharged, patients were advised to continue functional exercise, anticoagulant therapy, and timely reexamination.

### 2.3. Observation Index

1. The decrease of hemoglobin at 24 hours, 36 hours, and 48 hours after treatment.
2. The total postoperative blood loss and the maximum reduction of hematocrit (HCT).
3. The ROM of knee joint was studied before treatment, 6 months after treatment, and 12 months after treatment.
4. The scores of Fugl-Meyer motor function scale (FM-B) were studied before treatment, 6 months after treatment, and 12 months after treatment. In the FM-B scale, there were seven items: unsupported sitting position, healthy side spreading reaction, affected side spreading reaction, standing under support, standing without support, standing on healthy side, and standing on affected side [17]. The score of 0–2 for each item was scored according to three levels and a score of 0 to 14 indicated that the balance function was impaired. The lower the score, the more serious the balance dysfunction.
5. The scores of the Berg balance scale (BBS) were studied before treatment, 6 months after treatment, and 12 months after treatment. The score of BBS scale ranged from 0 to 56 and the higher the score, the stronger the balance ability [18]. From 0 to 20, the balance function was poor, the patient needs to ride in a wheelchair; 21 : 40 indicated a certain balance ability, the patient can walk with assistance; 41–56 indicated the balance function was better, the patient can walk independently. A score of less than 40 indicated the risk of falling.

### 2.4. Statistical Analysis

The research data were statistically analyzed by SPSS24.0 software, and the data of normal distribution were expressed by mean ± standard deviation and accepted independent sample *t* test. The counting data were tested by chi-square test and the grade data were tested by the Fisher exact method.

## 3. Results

### 3.1. The Decrease of Hemoglobin at 24 Hours, 36 hours, and 48 hours after Treatment

As indicated in Table 1, the decrease of hemoglobin in the study group at 24 hours, 36 hours, and 48 hours after treatment was lower compared to that of the control group (*P* < 0.05, Table 1).

The article "Safety and Efficacy of Single Condylar Knee Prosthesis When Treating Knee Single Compartment Osteoarthritis: A Prospective, Case-Randomized Controlled Study" was published in 2022. Journal: Comput Intell Neurosci.

### 3.2. The Total Blood Loss and Maximum Reduction of HCT after Operation

As indicated in Table 2, the total postoperative blood loss and the maximum reduction of HCT in the study group were remarkably lower (*P* < 0.05).

### 3.3. The ROM of Knee Joint Was Studied before Treatment, 6 months after Treatment, and 12 months after Treatment

As indicated in Table 3, ROM of the knee joint at 6 and 12 months after treatment in the study group was remarkably higher than that before treatment and remarkably higher compared to that of the control group (*P* < 0.05).

### 3.4. The Score of FM-B Scale before Treatment, 6 months after Treatment, and 12 months after Treatment

The FM-B scale scores of the study group after 6 months and 12 months of treatment were remarkably increased compared with those before treatment and were remarkably higher compared to those of the control group (*P* < 0.05, Table 4).

### 3.5. The Score of BBS Scale before Treatment, 6 months after Treatment, and 12 months after Treatment

After 6 months of treatment, the BBS scale scores of the study group after 12 months of treatment were remarkably increased compared with those before treatment and higher compared to the control group (*P* < 0.05, Table 5).

## 4. Discussion

Knee single compartment osteoarthritis is a chronic degenerative joint lesion [19]. At present, the number of patients with knee osteoarthritis in single compartment is increasing year by year and the incidence rate is high. According to statistics, the prevalence rate of people over 60 years old is 49%. The prevalence rate of people over 75 years old is as high as 80% [20]. Currently, the incidence of knee single compartment osteoarthritis is increasing year by year, which may become the fourth largest factor leading to disability by 2020 [21].

For patients with knee osteoarthritis, there are not many clinical methods that can be taken, mainly to reduce the weight-bearing and activity of the joint to delay the progress of the disease [22]. Early use of nonresidual drugs to control or alleviate the symptoms of patients, oral drugs involved in cartilage metabolism to prevent the progression of the disease. In clinical practice, it is considered that total knee prosthesis replacement and single condylar knee prosthesis replacement are effective methods for the treatment of single compartment osteoarthritis. The clinical application of total knee prosthesis replacement is long. The prosthesis design and operation technology are perfect, it can effectively relieve pain, restore function, and the survival rate of prosthesis is high. However, the pain-sensitive areas of some patients' knee joint are located on the medial side and the imaging findings are only unilateral compartment lesions of the knee joint. Therefore, with the continuous progress of artificial joint materials, design and surgical techniques, condylar knee prosthesis replacement has been applied to a certain extent when treating patients with knee osteoarthritis. Single ankle replacement for knee joint single compartment osteoarthritis has been favored by the majority of knee surgeons because of its obvious advantages and characteristics, such as less surgical trauma, short operation time and hospital stay, low hospitalization cost, satisfactory short-term effect, and so on. Riddle et al. reported that the number of American condylar knee prosthesis replacement increased by an average of 32.5% per year from 1998 to 2005 [23]. More and more researchers have believed that condylar knee arthroplasty can relieve pain and improve the quality of life of patients with osteoarthritis in single compartment, especially in medial compartment [24–32]. Therefore, a prospective, case-randomized controlled study was conducted to study the safety and efficacy of unicondylar knee prosthesis when treating knee single compartment osteoarthritis.

The article "Safety and Efficacy of Single Condylar Knee Prosthesis When Treating Knee Single Compartment Osteoarthritis: A Prospective, Case-Randomized Controlled Study" was published in 2022. Journal: Comput Intell Neurosci.

The results showed that the decrease of hemoglobin HB in the study group at 24 hours, 36 hours, and 48 hours after treatment was lower compared to that of the control group. The total blood loss and the maximum reduction of HCT in the study group were lower. The ROM of the knee joint in the study group at 6 and 12 months after treatment was remarkably higher than that before treatment and remarkably higher compared to the control group. The scores of FM-B scale and BBS scale in the study group at 6 and 12 months after treatment were remarkably higher than those before treatment and were remarkably higher compared to the control group. This study has shown that single condylar knee prosthesis is more safe and more effective when treating knee single compartment osteoarthritis. Additionally, it is more beneficial to reduce trauma, reduce perioperative blood loss, and improve the exercise and balance ability of patients.

Compared with total knee prosthesis replacement, single condylar knee prosthesis replacement has unique advantages: The main results are that the conventional choice of single condylar knee replacement is to use the lower limb fixator to suspend the lower limbs of the replacement side to facilitate the gap measurement. The release and balance of soft tissues is not emphasized, so there is no need to release the collateral ligament. The whole joint is more stable, the movement function is better, it is more conducive to the recovery of motor function and improve the balance ability of the limb. Second, the proprioceptive sensation of the joint can be close to normal to the maximum extent. Then, only a small amount of osteotomy is performed in the lesion compartment and sufficient bone mass is retained for possible secondary revision surgery. The effect of revision is similar to that of the primary total knee prosthesis replacement [33]. Lastly, functional exercises should be carried out earlier because of small incision, less bleeding, and less postoperative complications. 30 patients (32 knees) were followed up for an average of 53 months, of which 21 patients had polyethylene wear and only 2 patients needed revision surgery, and the thickness of polyethylene exceeded that of 10 mm [34]. Berger et al. followed up 51 patients (62 knees) with single condylar replacement with bone cement type of knee joint [35]. Taking revision or imaging prosthesis loosening as the standard, the 10-year survival rate was 98% and the 13-year survival rate was 95.7%. Swienckowski et al. reported 41 patients (46 knees) with single condylar replacement of knee joint, whose 11-year survival rate was 92% [36]. Hopper GP et al. have indicated that patients undergoing unicondylar knee prosthesis replacement have a higher quality of life than patients with total knee prosthesis replacement, specifically in 96.7% of patients who can participate in sports activities, while only 63.3% of patients with total knee prosthesis replacement [37]. In 1988, Mac Kinnon et al. reported that the 57-month survival rate of knee unicondylar replacement was about 95% [38]. In 1998, Murray et al. reported that the 10-year survival rate after knee joint unicondylar replacement was about 98% [39]. In 2004, Naudie et al. reported that the 5-year and 10-year survival rates after unicondylar knee replacement were 94% and 90%, respectively [40]. Romanowski et al. performed 13 cases of single condylar replacement with small incision, and the survival rate of 8-year follow-up was 93% [41]. Argenson et al. basically agree with these views through research and they believe that computer-aided systems will also increase the accuracy of surgery in the future [42]. Therefore, it can be considered that unicondylar knee prosthesis replacement has the advantages of high efficacy and safety when treating knee single compartment osteoarthritis. There are some limitations in this study. First, the sample size of this study is not large and it is a single-center study, so bias is inevitable. In future research, we will carry out multicenter, large-sample prospective studies, or more valuable conclusions can be drawn.

The article "Safety and Efficacy of Single Condylar Knee Prosthesis When Treating Knee Single Compartment Osteoarthritis: A Prospective, Case-Randomized Controlled Study" was published in 2022. Journal: Comput Intell Neurosci.

To sum up, the unicondylar knee prosthesis is safer and more effective in the treatment of noncompartmental osteoarthritis of the knee, facilitating less trauma and perioperative blood loss and enhancing the patient's motion and balance.

## Figures and Tables

**Figure 1:** Technology roadmap.

**Table 1:** The decrease of hemoglobin at 24 h, 36 h, and 48 h after treatment.

Grouping	After treatment 24 h (g/L)	After treatment 36 h (g/L)	After treatment 48 h (g/L)
Control group (*n* = 40)	13.54 ± 2.19	24.82 ± 3.11	36.99 ± 4.08
Study group (*n* = 40)	8.35 ± 1.12	15.69 ± 2.23	19.24 ± 3.02
*χ * ^2^ value	13.344	15.088	22.116
*P* value	<0.05	<0.05	<0.05

**Table 2:** The total blood loss and the maximum reduction of HCT after operation.

Grouping	Total postoperative blood loss (ml)	Maximum HCT reduction (%)
Control group (*n* = 40)	381.54 ± 105.19	0.05 ± 0.02
Study group (*n* = 40)	191.38 ± 75.12	0.03 ± 0.01
*t* value	9.304	5.567
*P* value	<0.05	<0.05

**Table 3:** The ROM of knee joint before treatment, 6 months after treatment, and 12 months after treatment.

ROM of the knee joint	Before treatment	Treatment for 6 months	Treatment for 12 months
Control group (*n* = 40)	105.82 ± 12.11	109.12 ± 9.39^*∗*^	113.19 ± 8.25^*∗*^
Study group (*n* = 40)	105.69 ± 12.03^*∗*^	118.14 ± 11.44^*∗*^	126.23 ± 8.35^*∗*^
*t* value	0.048	3.855	7.026
*P* value	0.962	<0.05	<0.05

^*∗*^represents that the 6-month and 12-month treatment in this group were compared with those before treatment, *P* < 0.05.

**Table 4:** The scores of FM-B before treatment, 6 months after treatment, and 12 months after treatment.

FM-B scale score (points)	Before treatment	Treatment for 6 months	Treatment for 12 months
Control group (*n* = 40)	7.52 ± 1.12	9.24 ± 0.22^*∗*^	11.29 ± 0.64^*∗*^
Study group (*n* = 40)	7.49 ± 1.09	11.08 ± 0.13^*∗*^	13.71 ± 0.15^*∗*^
*t* value	0.121	45.539	23.284
*P* value	0.904	<0.05	<0.05

^*∗*^represents that the 6-month and 12-month treatment in this group were compared with those before treatment, *P* < 0.05.

**Table 5:** The scores of BBS before treatment, 6 months after treatment, and 12 months after treatment.

BBS scale score (points)	Before treatment	Treatment for 6 months	Treatment for 12 months
Control group (*n* = 40)	30.23 ± 2.37	42.09 ± 2.47^*∗*^	46.59 ± 2.32^*∗*^
Study group (*n* = 40)	30.18 ± 2.42	49.25 ± 1.01^*∗*^	53.36 ± 1.14^*∗*^
*t* value	0.093	16.969	16.564
*P* value	0.926	<0.05	<0.05

## Data Availability

The datasets used and analyzed during the current study are available from the corresponding author upon reasonable request.
